The article "Integrated Design and Development of Intelligent Scenic Area Rural Tourism Information Service Based on Hybrid Cloud" was retracted in 2023. Reasons: unreliable results or conclusions; concerns about the data; concerns about the peer review; concerns about the citations.

# Integrated Design and Development of Intelligent Scenic Area Rural Tourism Information Service Based on Hybrid Cloud

**DOI:** 10.1155/2022/5316304

**Published:** 2022-06-16

**Authors:** Hong Zhang, Mingyang Li

**Affiliations:** Business School, Dalian University of Foreign Languages, Dalian 116044, China

## Abstract

Although the “Internet+” technologies (big data and cloud computing) have been implemented in many industries, each industry involved in rural tourism economic information services has its own database, and there are still vast economic information resources that have not been exploited. Z travel agency through rural tourism enterprise third-party information services and mobile context-awareness-based Z travel has achieved good economic and social benefits by deep value mining and innovative application of the existing data of the enterprise through the third-party information service of rural tourism enterprises and mobile context-aware travel recommendation service. It clearly demonstrates that, in order to maximise the benefits of economic data, rural tourist businesses should focus not only on the application of new technologies and methodologies but also on the core of demand and data-driven and thoroughly investigate the potential value of current data. This paper mainly analyzes the problems related to how rural tourism can be upgraded under the smart tourism platform, with the aim of improving the development of China's rural tourism industry with the help of an integrated smart tourism platform, and proposes a hybrid cloud-based integrated system of smart scenic rural tourism information services, which can meet the actual use needs of rural tourism, with good shared service effect and platform application performance, and promote the development of rural tourism and resource utilization rate.

## 1. Introduction

The rise of the smart tourism model provides a new opportunity for rural tourism information construction, and the full integration of rural tourism information technology and smart tourism development is beneficial to the realization of rural tourism industry development systemic linkage, but also the future of rural tourism economic construction indispensable main content, to enhance the impact of rural tourism, has important significance [1–3].

International rural tourism information technology started earlier, and in the late 1990s, some developed countries have formed the prototype of intelligent tourism. With the improvement of the level of information development and the popularization of intelligent technology, intelligent tourism development has become the main form of rural tourism development in some international developed countries.

The article "Integrated Design and Development of Intelligent Scenic Area Rural Tourism Information Service Based on Hybrid Cloud" was retracted in 2023. Reasons: unreliable results or conclusions; concerns about the data; concerns about the peer review; concerns about the citations.

Among them, the customised service model [4, 5], which analyses the market demand of tourism consumers to develop tourism programs and carry out the entire process of tourism management services from the perspective of consumers, effectively improving the accuracy of the positioning of the rural tourism industry and providing a strong guarantee for the expansion of potential consumer groups, is widely used in the development of intelligent tourism in Western Europe. In contrast to developed countries in Western Europe, the use of intelligent tourism technology in the development of rural tourism information technology in some North American countries is primarily reflected in the fields of marketing advertising and advertising information propaganda, with the use of information technology and intelligent technology in rural tourism services being relatively limited. This difference is mainly due to the different economic development patterns and economic development systems in different regions, so that each region must choose the appropriate way to carry out rural tourism informatization construction based on its own conditions, thus promoting the formation of a diversified rural tourism informatization development pattern worldwide. China's domestic rural tourism information construction started nearly 20 years later than the international developed countries, the early stage of development level is particularly lagging behind, and development resources are limited to economic development areas. Rural tourism informatization development has become the basis of modern rural tourism economic construction in China, influenced by the level of information technology development and the soft power of information management, especially in Central China, South China, and Southwest China, where rural tourism informatization development is relatively high. It is due to the development of information technology and the wide application of Internet technology that China's information-based rural tourism construction was formed with local characteristics and cultural style. With the launch of many domestic tourism apps in recent years, the development of rural smart tourism has gradually been emphasized by all regions and has become a major thrust for regional economic development. Although China's current rural intelligent tourism development is relatively good, there are still some basic problems to be solved, which is also an important factor hindering the development of China's rural tourism information construction [6, 7]. The basic features of cloud computing are shown in Figure 1.

China and governments at all levels have deployed the rural revitalization strategy, and rural revitalization has become an important grasp of China's three agricultural works during the period of China's rural transformation and development. Economic revitalization is the foundation of rural revitalization, and rural tourism industry has become an important way to promote rural economic revitalization and industrial prosperity because of its diversified resource elements input requirements to integrate rural natural ecology and traditional culture and plays a pivotal role in the transformation of modern rural production mode and industrial structure. And with the development of modern technologies such as big data and Internet of Things, rural tourism development has advanced with the times, through the deep integration of technology and tourism, not only to achieve the systematic integration of tourism resources but also through the application of big data, cloud computing, artificial intelligence technology, etc. [8, 9], to improve tourism infrastructure, enhance tourism experience, and promote services with technology, forming a new tourism industry of wisdom, information, and personalization and creating a wisdom tourism. With the help of wisdom tourism-related technology and production and management system, we improve the rural tourism service system, consolidate the technical foundation of rural tourism development, promote the construction of tourism-oriented villages with wisdom tourism, realize rural affluence, rural income, and ecological improvement with the new mode of tourism industry development, and provide the industrial foundation for comprehensive rural revitalization. This paper focuses on the overall architecture of the wisdom tourism hybrid platform and proposes a hybrid cloud-based integrated architecture of wisdom scenic rural tourism information service, which realizes the virtualization management of rural tourism resources through cloud computing to achieve unified sales, service, and management of rural tourism resources. As an important service industry, exploring a cloud computing application scheme suitable for rural tourism scenic areas is an important element of future smart tourism construction. The deployment strategy of hybrid cloud is analyzed, and the effectiveness of the method in this paper is verified through experiments.

The article "Integrated Design and Development of Intelligent Scenic Area Rural Tourism Information Service Based on Hybrid Cloud" was retracted in 2023. Reasons: unreliable results or conclusions; concerns about the data; concerns about the peer review; concerns about the citations.

The following is the paper's organization paragraph: Section 2 discusses the related work. The suggested work's approaches are examined in Section 3. The trials and results are discussed in Section 4. Finally, the research job is completed in Section 5.

## 2. Related Work

### 2.1. Rural Intelligent Tourism Construction

There will very certainly be a lot of infrastructure rehabilitation and industrial development as part of the process of rejuvenating the countryside and boosting rural tourism. To avoid destroying the original rural landscape and cultural traditions during construction and development, intelligent tourism technology can be used to achieve sustainable utilization, such as using mapping and positioning technology in intelligent tourism, applying satellite remote sensing mapping, drone mapping, tilt photography technology, and Baidoo precise positioning technology in large regional project implementation monitors. In terms of monitoring regional project implementation, land resource protection, and use, as well as environmental protection of rural villages and restoration of ancient buildings, tourism development and utilization can be realized without changing the original rural landscape, and the authenticity of tourism resources can be protected as much as possible. For the intangible cultural heritage, mainly intangible cultural heritage, which is widely inherited in the countryside, big data technologies such as database, knowledge mapping, block chain, and other technologies in smart tourism can be used to achieve sustainable utilization of traditional rural culture. The purpose of wisdom tourism development for rural tourism system construction is to carry out scientific wisdom tourism development management layout according to the characteristics of rural tourism information development, promote the diversified design of wisdom tourism content [10–13], and develop wisdom tourism strategies centered on rural tourism development. For example, vigorously promote rural tourism with some companies to enhance tourism market resources to rural tourism construction, using joint development with relevant enterprises to achieve the synchronization of rural tourism and wisdom tourism development content, so that rural tourism information construction can benefit from mobile Internet for effective information promotion. On the one hand, to meet the basic needs of rural tourism informatization construction; on the other hand, to improve the perfection of industrial content of wisdom tourism development, so that rural tourism informatization development and wisdom tourism industry layout can effectively achieve mutual benefit and win-win situation. To strengthen rural tourism informatization of wisdom tourism synergistic development mainly tourism development marketing, service management and tourism project design, and other levels to achieve synergistic development and wisdom tourism as a carrier to rural tourism service information conduction, the process of rural tourism informatization construction mainly plays a terminal service management role, that is, to achieve offline tourism services and management planning [14–17]. Rural tourism information development background and intelligent tourism industry integration should give rural tourism certain help in tourism development innovation. For example, in travel mode, travel items and travel content can be adjusted according to the needs of travel consumer groups. Through the smart tourism data platform and information management, it is possible to ensure that the content of tourism projects and publicity content remain unified, so that the construction of rural tourism information and the integration of smart tourism can ensure a consistent pace, keep pace with the times [18], and promote industrial construction and development.

The article "Integrated Design and Development of Intelligent Scenic Area Rural Tourism Information Service Based on Hybrid Cloud" was retracted in 2023. Reasons: unreliable results or conclusions; concerns about the data; concerns about the peer review; concerns about the citations.

### 2.2. Hybrid Cloud

The industry has progressed from simple computing virtualization to the cloud of the entire data center, employing a software-defined approach to automate and scale the administration of computing, network, and storage resources in the data center. A multi-AZ interoperable resource sharing paradigm has been adopted across various cloud data centers by large companies with numerous data centers. Today, an increasing number of businesses are combining clouds from various providers to solve specific business concerns. The evolution from traditional IT to the cloud has given birth to a large number of different cloud technologies (see Figure 2) [19–21]. The most basic categories include traditional IT environments, private clouds built by enterprises, hosted clouds built by service providers for specific enterprises, and public clouds built by service providers for the general public. Each production environment in turn has different technology choices and feature options, both large and small, framing an exceptionally complex application deployment relationship. In the short and medium term, different enterprises and different applications have their own intrinsic reasons for choosing different execution environments and cannot simply choose one and discard the others.

At this stage, enterprises usually use three types of computing resources, namely, dedicated server resources running in enterprise data, virtual resource pools established on the basis of private clouds in enterprise data centers, and computing resources provided by public cloud providers [22]. For these three different types of enterprise computing resources, it is less cost-effective to use a private cloud that consumes a lot of resources to run enterprise applications that would be more efficiently run on a public cloud platform, but some enterprise-critical applications must be run in a private cloud environment. The advantage of hybrid cloud is that it can adapt to the needs of enterprises for different platforms, providing both the security and convenience and management and operation and maintenance levels of a private cloud and the openness and convenience of a public cloud, and is now considered to be the mainstream business cloud solution that enterprises will increasingly adopt in the future. These platforms operate independently of each other and are interconnected, allowing data to be shared as required to meet service agreements [23]. Deploying a successful hybrid cloud starts with a good understanding of which datasets and applications are best suited to run in a private cloud environment and which can be delivered to a trusted cloud service provider to ensure that a fully integrated platform can be provided to the enterprise. A trusted partner can help identify and articulate the reasons for a well-performing business, in addition to helping oversee a catalog of service portfolios, including creating metrics and portfolio management. Finally, the partner can help select a portfolio of services for delivery models such as financial, compliance, security, and workload. The specific hybrid cloud deployment strategy is shown in Figure 3.

The article "Integrated Design and Development of Intelligent Scenic Area Rural Tourism Information Service Based on Hybrid Cloud" was retracted in 2023. Reasons: unreliable results or conclusions; concerns about the data; concerns about the peer review; concerns about the citations.

## 3. Methodology

### 3.1. Hybrid Cloud Platform Architecture Design

Both public and private clouds offer infrastructure resources including processing, storage, and networking, as well as open APIs for consumers to employ. However, each cloud provider's APIs are distinct, and there is no consistent standard, which makes adapting heterogeneous clouds a difficult task for customers. Therefore, in this paper, we build independent Kubernetes container clusters in each cloud provider, such as public and private clouds, and then design and implement a unified global controller to manage and schedule the Kubernetes container clusters on each heterogeneous cloud at the upper layer. This ensures API homogeneity across the underlying heterogeneous clouds, as well as the simplicity of cross-cloud deployment, migration, and business elastic scalability.  Figure 4 depicts the full hybrid cloud platform architecture.

The hybrid cloud management platform mainly manages application publishing and resource scheduling of container clusters on the underlying heterogeneous cloud and contains four modules: API, scheduler, controller, and database. The API is mainly used to receive commands from the front-end, the scheduler is used to schedule Kubernetes clusters in the heterogeneous cloud, the controller is used to handle business logic, and the database is used to persistently store resource data managed by the platform. The underlying public or private cloud Kubernetes cluster mainly manages the scheduling and dispatching of resources of a single container cluster, including master and node nodes. Master mainly controls the resource scheduling of a single cluster, and node runs the actual business container as a working node.

The article "Integrated Design and Development of Intelligent Scenic Area Rural Tourism Information Service Based on Hybrid Cloud" was retracted in 2023. Reasons: unreliable results or conclusions; concerns about the data; concerns about the peer review; concerns about the citations.

### 3.2. Heterogeneous Kubernetes Access Design

To deploy Kubernetes on each heterogeneous cloud infrastructure of the user, the upper global controller needs to add the platform address, port and Barberton of each Kubernetes cluster, etc. The upper controller makes calls through the standard API and the underlying Kubernetes. Namespaces of Kubernetes represent namespaces, which are mainly used to achieve resource isolation of tenants. Nodes represent host nodes in the cluster, which are the bearers of resource scheduling. Deployments are primarily used to manage the number of copies of applications. Pods are the smallest units for application operation and scheduling. Services are services that can expose access portals for back-end applications.  Figure 5 depicts a schematic diagram of cloud data transfer and exchange.

### 3.3. Hybrid Cloud Framework Application Performance Analysis

Considering the economic cost and time cost, often different cloud service models are used to accomplish big data analysis. Therefore, the hybrid cloud platform should give the estimated computational resources and computation time to the user before the user submits the data with the target problem to determine the required virtual machine configuration. Initially, the MapReduce application is deployed on *N* internal private cloud VMs, and all the initial invariant data is stored in a distributed manner. When there are *M* external public cloud VMs scaled to support *N* internal VMs for big data analytics tasks, the perception policy rescales the deployment of MapReduce applications and iterates the MapReduce-based big data analytics application on the generated hybrid cloud platform. For analysis, let the internal VMs have the same configuration capability as external VMs, and users can trace the historical state of the application or have access to the following MapReduce performance metrics: the total number of map/reduce tasks, denoted as PM and PR; the number of physical slots for performing map/reduce tasks, denoted as kM and kR; the average time to execute map, reduce, and scheduling tasks, denoted as AM, AR, and AS; and the average amount of scheduling data per execution of map, reduce, and scheduling tasks, denoted as DM, DR, and DS. In addition, let the dynamic behavior of the big data analysis application at runtime be measurable; i.e., the first iteration process is known a priori, while the input data volume, newly generated data volume, and computational complexity during each subsequent MapReduce operation are independent of each other. The internal virtual machine performance evaluation metrics are used in the *i*^th^ map operation, and the set of tasks with the number Num_*M*,*i*_ is assigned to *k*_*M*,*i*_ physical machines using a greedy allocation strategy. In this process, the task scheduling operation needs to be started first, so extra time is introduced and its time overhead needs to be considered separately, and its execution time is noted as *T_1_*, whose value is related to the physical device performance and software system working mechanism, and can be considered as a constant. The theoretical lower bound on the execution time of subsequent task execution occurs in the case that the slowest task is scheduled to be executed last, while the previous Num_*R*,*i*_ tasks have already been executed. Therefore, the theoretical maximum execution time of the *i*^th^ map operation is

(1) $$\begin{array}{c} T_{M\dot{,i}}^{\max}=\frac{\left(\text{Nu}{\text{m}}_{M_{i}}-2\right)\bar{\tau }}{k_{M,i}}+\tau_{\max}, \end{array}$$

where *τ* is now the average execution time of the task and *τ*_max_ is the slowest execution time of the task. Further, its minimum execution delay occurs when the workload is fully balanced, and all tasks are executed with normal efficiency. Therefore, the theoretical minimum execution time of the *i*^th^ map operation as

(2) $$\begin{array}{c} T_{M_{-}}^{\min}=\frac{\left(\text{Nu}{\text{m}}_{M_{-}}-1\right)\bar{\tau }}{k_{M_{\dot{i}}}}. \end{array}$$

Since the reduce and map operations in MapReduce are independent of each other but do not require task scheduling operations again, the minimum and maximum execution times for the *i*^th^ reduce operation are

(3) $$\begin{array}{c} \left\{\begin{array}{c} T_{R_{-}}^{\max}=\frac{\left(\text{Nu}{\text{m}}_{R_{\dot{i}}}-1\right)\bar{\tau }}{k_{R_{-}}}+\tau_{\max},\\ T_{R_{-}}^{\min}=\frac{\text{Nu}{\text{m}}_{R_{\dot{-}}\bar{\tau }}}{k_{R_{\dot{H}}}}, \end{array}\right. \end{array}$$

where *T*_*R*_−__^max^ and *T*_*R*_−__^min^ are the theoretical upper and lower bounds of the execution time of the *i*^th^ reduce operation, Num_*M*,*i*_ is the number of tasks in the *i*^th^ reduce operation, and *k*_*R*,*i*_ is the number of physical machines in the *i*^th^ reduce operation. In summary, for the *i*^th^ iteration process, the lower bound on the time delay required to complete its execution can be estimated by the following equation

(4) $$\begin{array}{c} T_{i}^{\max}=T_{M_{-}}^{\max}+T_{R_{-}}^{\max}+T_{1}. \end{array}$$

For a big data analysis application with iteration *I*, the total completion time can be estimated by the following equation.

(5) $$\begin{array}{c} T^{\max}=\overset{I}{\underset{i=1}{\sum }}\;\left(T_{M_{-}}^{\max}+T_{R_{-}}^{\max}\right)+IT_{1}. \end{array}$$

The article "Integrated Design and Development of Intelligent Scenic Area Rural Tourism Information Service Based on Hybrid Cloud" was retracted in 2023. Reasons: unreliable results or conclusions; concerns about the data; concerns about the peer review; concerns about the citations.

### 3.4. Rural Tourism Information Ranking

Let the length of all retrieval result lists be *N*. The rating of the *i*^th^ data in the list is (*N* − *i* + 1), so the first data in the retrieval result list with the highest rating can be obtained as *N* and the last data with the lowest rating. Assuming that a data appears more times in different retrieval result lists, the rating of the data can be expressed as the sum of the rating values of each retrieval queue. Then, the data that appears in all of the multiple retrieval result lists has a higher rating than the one that appears individually. The total score is obtained by first scoring each retrieval result data, and then, the data appearing in different retrieval result queues are summed into a list and sorted according to the weight value from largest to smallest. Let *MM* be the amount of data in the longest retrieval return list. In this paper, the longest retrieval chain is *NC*, i.e., *MM* = *MO*. For the *j*-th retrieval result list, let the rating base be *W*_*j*_, and let the rating of the *i*^th^ data in the *j*-th column be *W*_*j*_*∙*(*MM* − *i* + 1). The relevance of the search term to its corresponding search category *C* and the amount of data in the retrieval queue will have an impact on the scoring base *W*_*j*_. The retrieval queue scoring base *W*_*j*_ is shown as follows:

(6) $$\begin{array}{c} W_{j}={\mathrm{rank}}_{C}\cdot \sqrt{{\text{sim}}_{C}}\cdot {\text{num}}_{C}, \end{array}$$

where assuming the best similarity between retrieval category *C* and retrieval keywords, rank_*C*_ is 1. In the second rank,rank_*C*_is 0.5, and in the third rank,rank_*C*_is 0.25.sim_*C*_ is Sim(*q*, *c*), and num_*C*_ indicates the number of data in the retrieval list. If a retrieval result list is not summed by retrieval category, rank_*C*_ is 0.5 and sim_*C*_ is 0.1.

### 3.5. Realize Off-site Disaster Recovery

A new private cloud data center is built off-site, and public cloud services are rented to form a “hybrid cloud” architecture. At the same time, the local data center of the health Bureau is used as the disaster recovery center, which eventually forms a “hybrid cloud” based two-location, three-center architecture. The existing hardware and network resources are fully protected, and under the cloud environment of the new data center, the appropriate level of protection is provided for each level of business, and the colocation and off-site disaster recovery of business and data backup are completed. The core key services of the new private cloud data center are built in 1 : 1 mode, which can realize business-level disaster recovery, and when the main system fails, the backup system takes over the business without losing business data. In addition, in order to avoid the hidden danger of data loss caused by natural disasters, the local server room of the health Bureau is used as the disaster recovery center, and a flexible deployment backup strategy is adopted, so that when the private cloud data center fails, no data can be lost, storage level disaster recovery can be realized, and the local data center has the ability to quickly resume business. The hybrid cloud disaster recovery solution is shown in Figure 6.

The article "Integrated Design and Development of Intelligent Scenic Area Rural Tourism Information Service Based on Hybrid Cloud" was retracted in 2023. Reasons: unreliable results or conclusions; concerns about the data; concerns about the peer review; concerns about the citations.

## 4. Experiments and Results

### 4.1. Dataset

In order to verify the effectiveness of the algorithm proposed in this paper, cross-simulation tests are conducted. The user's rural tourism retrieval records were all divided into 10 subsets, each with the same number of tourism retrieval records. The retrieval algorithm was repeated 10 times for each different subset of data, and 9 of them were used as the training set. For the training set, the matrix DT_train_ and matrix DC_train_ are built using the method proposed in this paper, and the matrix DT_test_ and matrix DC_test_ are built according to the test set. Once the individual retrieval feature matrix *M* is constructed, the relevance of the retrieval categories in the DT_test_ matrix and DC_test_ matrix to the retrieval keywords is obtained, and the relevance score is performed. The experiments are from a travel information website, and the statistical results are shown in Table 1.

### 4.2. Experimental Results

For each user's retrieval, the algorithm feeds the user 3 categories with high relevance to the retrieved term, and the following equation is used to score the relevance of the retrieved category to the retrieved keyword.

(7) $$\begin{array}{c} \begin{array}{c} \text{Accuracy}=\frac{\sum_{\text{Cletop }3}\text{ scor}{\text{e}}_{ci}}{n},\\ {\text{score}}_{ci}=\frac{1}{1+{\mathrm{rank}}_{ci}-\text{ideal}\_{\mathrm{rank}}_{ci}}, \end{array} \end{array}$$

where *n* denotes the number of all retrieval categories related to the retrieved keywords, score_*ci*_ denotes the rating of the top three retrieval categories *ci* in terms of relevance. rank_*ci*_ denotes the ranking of retrieval categories *ci*, and ideal_rank_*ci*_ denotes the highest ranking that retrieval categories ci may receive. The feature matrix simulation experiments use the Rocchio algorithm and the Im-Rocchio algorithm proposed in this paper to calculate the user retrieval feature matrix *M*, respectively, and then, use the user retrieval feature matching algorithm to perform category matching and calculate the matching accuracy. From the results in Table 2, we can see that the average retrieval accuracy of the Im-Rocchio algorithm proposed in this paper is higher than that of the standard Rocchio algorithm.

The article "Integrated Design and Development of Intelligent Scenic Area Rural Tourism Information Service Based on Hybrid Cloud" was retracted in 2023. Reasons: unreliable results or conclusions; concerns about the data; concerns about the peer review; concerns about the citations.

Feature matching simulation experiments are first conducted using the experimental dataset to compare user retrieval feature matching, generic retrieval feature matching, and 3 kinds of mixed feature threshold extraction matching, and the average accuracy of retrieval results is counted, as shown in Table 3. From the results in Table 3, we can see that the precision of the three-hybrid feature threshold extraction matching algorithms is not much different, but all of them are more precise than the user retrieval feature matching and universal retrieval feature matching, so the hybrid feature threshold extraction matching algorithm is better than the other algorithms. In addition, user retrieval feature matching is better than generic retrieval feature matching. To further validate the performance of the algorithm, the hybrid feature threshold extraction matching algorithm is considered and the training set is gradually increased. The above experiments show that when the data training set is small, the user retrieval feature matching algorithm is less accurate than the general-purpose retrieval matching algorithm. Even when the training set is small, the hybrid feature threshold extraction matching algorithm still achieves better results. When the training set is gradually increased, the accuracy of both the user retrieval feature matching strategy and the hybrid feature threshold extraction matching strategy increases.

### 4.3. Hybrid Cloud Performance Testing

In this experiment, the size of the input data volume used is 20 GB, and the size of the data volume processed by each mapping processor varies randomly, which equates to the number of mapping processors varying randomly. As a result, the following is the data sample creation process utilized to construct the random forest algorithm: First, HDFS is installed on three virtual machines in the internal virtual cloud and configured to generate data blocks using TestDFSIO. After the initial data is written, the HDFS deployed on the internal private cloud VMs can be further extended and deployed to the external public cloud VMs; second, during the load balancing phase, another TestDFSIO program is made to start at the same time. At the same time, at least one copy of each data block stored internally during the load balancing phase is moved to the externally deployed VMs. During the experimental run, the amount of data migrated to the external public cloud in the load balancing phase is recorded, thus forming a data sample containing different VM configuration scenarios and the performance of the corresponding algorithms. The proposed steps are then applied to construct a random forest. Denote the configuration scheme with *N* virtual machines deployed on the internal private cloud and *M* virtual machines deployed on the external public cloud as *N*-on-*M*-off. Let *M* = 0 denote the traditional single cloud storage scheme in the benchmark case, existing methods as a comparison, and *M* > 0 denote the proposed hybrid cloud storage scenario. The TestDFSIO experiments in the baseline and hybrid configuration scenarios are repeatedly executed 10 times, and these results are computed for the parameter *β*.  Table 4 gives the correspondence between the data transfer time and the load balancing time under the indicated partial configuration scenarios. Among them are configuration 1: 3-on-0-off; configuration 2: 3-on-3-off; configuration 3: 3-on-6-off; and configuration 4: 3-on-9-off. It can be seen that the hybrid cloud model, where the rack-aware policy-based data migration storage and load balancing significantly take up physical overhead, reduces concurrent read throughput, and the load balancing overhead time rises by more than 40.5 percent compared to the single cloud model.

The article "Integrated Design and Development of Intelligent Scenic Area Rural Tourism Information Service Based on Hybrid Cloud" was retracted in 2023. Reasons: unreliable results or conclusions; concerns about the data; concerns about the peer review; concerns about the citations.

## 5. Conclusion

The importance of rural tourism to rural revitalization is largely due to its high industrial correlation feature, which relates to transportation, accommodation, medical care, entertainment, catering, and a series of other supporting industries. Hybrid cloud platform has obvious technical and economic advantages because it combines the advantages of private cloud security and reliability and public cloud computing power. However, running intensive data businesses such as big data analytics under the hybrid cloud framework is still in its infancy, and there are difficulties in mismatching the underlying data storage with advanced applications and inaccurate application execution time prediction. The cloud platform is a new type of sharing infrastructure that employs cloud computing technology to gather a huge number of online resources and manages them automatically with software. The hybrid cloud-based integrated system of information services for rural tourism in smart scenic areas designed in this paper can use the hybrid cloud platform to get a large number of available resources in rural tourism and use software to manage them automatically. The test of this paper shows that the platform shares a relatively large number of resources and has comprehensive contents to meet the needs of users, and the rural tourism resources have good sharing application effects, which can improve the economic benefits of rural tourism.

The article "Integrated Design and Development of Intelligent Scenic Area Rural Tourism Information Service Based on Hybrid Cloud" was retracted in 2023. Reasons: unreliable results or conclusions; concerns about the data; concerns about the peer review; concerns about the citations.

## Figures and Tables

**Figure 1:** Map of the basic features of cloud computing.

**Figure 2:** Cloud computing trends.

**Figure 3:** Hybrid cloud deployment strategy flowchart.

**Figure 4:** Overall hybrid cloud platform architecture.

**Figure 5:** Sharing of data.

**Figure 6:** Hybrid cloud disaster recovery solution.

**Table 1:** Experimental dataset.

Statistics	Number of species	Query the records	Average record	Related documentation	Average kind	Different words
User 1	11	49	4.50	335	1.10	7965
User 2	09	52	6.10	168	01	6248
User 3	07	62	7.20	276	10	6689
User 4	08	49	5.20	103	1.20	4893
User 5	12	69	6.90	158	1.10	4903
User 6	09	39	4.50	164	01	4405
User 7	10	32	3.80	213	01	4498

**Table 2:** Accuracy comparison results.

Accuracy	User 1	User 2	User 3	User 4	User 5	User 6	User 7
Rocchio	0.65	0.71	0.89	0.72	0.81	0.70	0.69
Proposed algorithm	0.85	0.89	0.92	0.80	0.83	0.95	0.78

**Table 3:** Comparison of average accuracy of different algorithms.

Method	Personal characteristics match	Universal feature matching	Mixed feature matching 1	Mixed feature matching 2	Mixed feature matching 3
Accuracy	0.7658	0.9046	0.7051	0.9158	0.8957

**Table 4:** Average completion time per iteration of TestDFSIO.

Configuration serial number	Configure	Time per iteration/min	*β*
Configuration 1	3-on-0-off	6.90	3.40
Configuration 2	3-on-3-off	11.80	3.41
Configuration 3	3-on-6-off	11.90	3.38
Configuration 4	3on-9-off	11.60	3.45
Configuration 5	3-on-12-off	12. 05	3.42

## Data Availability

The datasets used during the current study are available from the corresponding author on reasonable request.
